# Multimodal MRI Analysis of Brain Metabolism in Maintenance Hemodialysis Patients Based on Cognitive Computing

**DOI:** 10.1155/2021/7231658

**Published:** 2021-08-09

**Authors:** Yan Zhang, Hui Ma, Xinguang Lv, Qinjun Han

**Affiliations:** ^1^Magnetic Resonance Room of Imaging Department, Baoji Hospital of Traditional Chinese Medicine, Baoji, Shaanxi 721001, China; ^2^Department of Radiology, Baoji Hi-Tech Hospital, Baoji, Shaanxi 721000, China; ^3^Foreign College of Baoji University of Arts and Sciences, Baoji, Shaanxi 721000, China

## Abstract

This paper investigates cognitive computation of brain metabolism in maintenance hemodialysis patients with multimodal MRI therapy assessment. This paper constructs a cross-individual emotion recognition method using dynamic sample entropy pattern learning. The cross-individual emotion recognition was carried out on subjects using the EEG emotion dataset SEED. The experimental results show that the proposed dynamic sample entropy-based pattern learning has better performance in cross-individual emotion recognition and exhibits better generalization and generalization ability when compared with the results of existing related studies. The constructed cognitive computing method for cross-individual emotion state recognition achieves optimization and innovation of EEG emotion pattern recognition, which can effectively predict people's mental emotion state from EEG signals. We also explore the value of diffusion-weighted magnetic resonance imaging and dynamic enhanced magnetic resonance imaging-based volumetric measurements in assessing the efficacy of neoadjuvant therapy in maintenance hemodialysis patients. We analyze and compare the results of different studies to find the best multimodal MRI to assess the efficacy of neoadjuvant therapy in maintenance hemodialysis patients. The use of ADC value growth rates to assess neoadjuvant efficacy provides the best diagnostic efficacy and allows the screening of patients who respond well to neoadjuvant therapy while avoiding the impact of two different b-value combinations commonly used to assess neoadjuvant efficacy.

## 1. Introduction

The specific pathogenesis of cognitive impairment in maintenance dialysis patients is not well understood, and possible mechanisms include vascular damage, toxin damage, and dialysis treatment factors. Among them, the mechanism of vascular injury plays an important role [1]. Dialysis patients have numerous risk factors associated with vascular injuries, such as hypertension, diabetes, hypercholesterolemia, advanced age, atherosclerosis, myocardial infarction, atrial fibrillation, and smoking, among the traditional risk factors. Also, the dialysis population has some risk factors specific to the normal renal function population, such as uremic toxins, inflammatory factors, endocrine hormones and vitamins, electrolytes, acid-base factors, and anemia, which may lead to vascular injury and also direct toxic damage to the central nervous system by modulating neurotransmitters, interfering with brain metabolism, damaging neurons, and affecting amyloid plaques, which may lead to cognitive dysfunction [2]. Dialysis treatment factors including dialysis case, frequency, and dialysate temperature may cause brain damage through hemodynamic fluctuations [3].

In recent years, with the continuous development of imaging technology and examination means of multimodal functional magnetic resonance, research, discovery, and results for the structure, function, and metabolism of the human brain have made amazing progress, which also provides more reliable techniques and methods for the study and diagnosis of end-stage renal disease patient-related encephalopathy such as cognitive dysfunction, and noninvasive neuroimaging technology provides a promising way to achieve these goals [4]. The use of noninvasive neuroimaging techniques has been increasingly applied to this disease to provide a reliable clinical basis for early diagnosis and delay of disease progression to the maximum extent possible [5]. The multimodal MRI ultrasound instrument transmits ultrasound beams to observe the changes in blood flow velocity, blood vessel distribution, and blood flow status of suspected diseased tissues and diagnoses tumors in combination with ordinary ultrasound images. Blood flow information, as auxiliary information for hemodialysis diagnosis, can improve its diagnostic accuracy. At the same time, multimodal MRI ultrasound examination has no harm to the patient's body and no pain in the examination process. It has been widely recognized and recognized in clinical applications in order to obtain the blood flow signal inside the blood [6].

This paper focuses on two aspects of auditory attention decoding and cross-individual mental-emotional state recognition, exploring cognitive computational methods and technical implementation of auditory target attention, auditory selective attention decoding and cross-individual mental-emotional state recognition, enabling effective prediction and inference of human mental attention and emotional states and accurate understanding of human auditory attention cognition and emotional intentions. Voxel-based morphometry is a new imaging technique for morphological measurement of magnetic resonance cranial images and automatic or manual quantitative or semiquantitative measurement of whole-brain volume at the voxel level, which allows the quantitative measurement and comprehensive and objective assessment of neuroanatomical changes in different groups of brains, such as abnormal changes in brain tissue structure, morphology, volume, density, or signal, with high accuracy and reproducibility. This paper is divided into five parts: the first part is the introduction, which introduces the background and significance of this paper and describes the research idea of this paper. The second part is the introduction of related work, which reviews and evaluates the current status of domestic and international research. The third part investigates the cognitive computation of brain metabolism and multimodal MRI in maintenance hemodialysis patients, from the extraction of relevant features of maintenance hemodialysis patients to the construction of cognitive computation models and then to the assessment of multimodal MRI therapy. The fourth part is the analysis of the results, which analyzes the value of the study in this paper. The fifth part is the conclusion and recommendations. It summarizes and analyzes the previous studies, makes recommendations, points out the main contributions of this paper, and indicates the limitations and prospects for future research.

## 2. Related Work

Emotion perception is one of the important signs of human intelligence, and people use emotional expression to convey information, understand their environment and current situation so that they can better adapt to various social interactions. Donahue et al. proposed a study of EEG emotion recognition combining EEG feature selection and kernel classifier. The study used a variety of EEG signal features-statistical features, band power at different frequencies, Horthy parameters, and fractal dimension, where statistical features included median, standard deviation, and kurtosis coefficient. The frequency bands of EEG signals were used, *θ* (4–8 Hz), low *α* (8–10 Hz), *α* (8–12 Hz), *β* (12–30 Hz), and *γ* (30–45 Hz), and then a mutual information-based feature selection method and a kernel classifier were used to optimize the performance of the emotion classification task [7]. Prado et al. proposed a combined machine learning model-based approach to automatically detect EEG emotional arousal, and their study evaluated in detail six machine learning models—Fisher's linear discriminator, support vector machines, artificial neural networks, classification trees, k-nearest neighbors, and plain Bayesian—were evaluated in detail for their emotion recognition performance. Synthesizing the existing research related to EEG emotion pattern recognition, machine learning as a typical representative of EEG emotion pattern learning and classification method is widely used in the research of EEG signal emotion recognition [8]. The classification algorithm of machine learning is used to classify and recognize the emotional features of EEG signals, and the task of emotional state recognition is realized from the EEG feature information [9].

Lin et al. used two methods, voxel-based diffusion tensor analysis and spatial statistical analysis based on fiber tract skeleton, to study brain white matter fibrils in ESRD patients, and found not only that there were multiple brain white matter areas with reduced FA values in the brains of ESRD patients, and some brain areas with reduced FA values were correlated with the duration of dialysis and cognitive function scores, and combined with ESRD patients' DTI abnormalities in the cerebral white matter further revealed the presence of high-risk factors leading to damage of cerebral white matter in ESRD patients, pointing out that different degrees of diffuse cerebral enema and comprehensive lesions of cerebral white matter demyelination are the main manifestations of cranial microstructure damage in ESRD patients [10]. In a study by Cai et al., it was found that ESRD patients undergoing routine hemodialysis had multiple areas of reduced FA and increased MD in the cranial brain. Areas of brain tissue with increased FA values, including the frontotemporal junction, corpus callosum knee, and fornix, suggesting that both patients with chronic renal insufficiency and ESRD patients in the middle to late stages can cause or even exacerbate degenerative brain changes associated with population aging, further revealing that ESRD patients with more than two risk factors for cardiovascular disease may be at high risk for accelerated damage to their cerebral white matter integrity and that ESRD hemodialysis patients are at high risk for developing stroke and cognitive dysfunction, and that microstructural and pathological alteration in cerebral white matter may be present in the early manifestations of these serious complications [11]. Hemodialysis is an invasive, lifelong treatment, and patients may experience new physical symptoms such as fatigue, pain, dry skin, itching, and sleep disturbances due to the disease itself or the treatment.

Cognitive dysfunction is a type of neurological impairment in maintenance dialysis patients with a high prevalence and may cause multiple adverse outcomes [12]. Its specific pathogenesis is still not well defined, and the mechanism of vascular damage may play an important role. Cerebrovascular disease is prominent in dialysis patients, and typical features of cerebral small vessel disease such as lacunar cerebral infarction, cerebral white matter hyperintensities, cerebral microhemorrhage, and cerebral atrophy may be closely associated with cognitive impairment. Atherosclerosis is a risk factor for cognitive impairment, and there is insufficient evidence that its noninvasive surrogates, including carotid intima-media thickness pulse wave velocity, are associated with cognitive impairment in dialysis patients. Lipid metabolism has significant implications for cardiovascular disease, and lipid metabolism disorders are prominent in dialysis patients, but there is an “inverse epidemiological phenomenon” with cardiovascular disease. It remains unknown whether the classical lipid components that affect cardiovascular events in the general population also contribute to the high incidence of cardiovascular events in dialysis patients and whether abnormal lipid metabolism is involved in the development of cognitive impairment in dialysis patients. The application of approaches may identify highly sensitive and specific markers of cognitive impairment in dialysis patients.

## 3. Cognitive Computing of Brain Metabolism in Maintenance Hemodialysis Patients with Multimodal MRI Study

### 3.1. Study on the Characteristics of Maintenance Hemodialysis Patients

The dimensions of fatigue in maintenance hemodialysis patients were significantly and negatively correlated with quality of life, and the more fatigued the patients were, the lower their quality of life was, and the behavioral dimension had the highest correlation coefficient among the four dimensions with a moderate correlation. The impact of maintenance hemodialysis fatigue on patients' quality of life is multifaceted. Fatigue reduces patients' ability to perform physical and mental activities, and many daily activities and tasks cannot be performed alone, and patients' roles and functions in family and society are changed, which ultimately affects the patient's quality of life [13, 14].

Physiological functions mainly reflect the patient's ability to perform activities of daily living, such as dressing, walking, walking upstairs, bending, and bathing. Patients have complications and physical pain, but they generally have different degrees of self-care ability. Most of the young and middle-aged patients and patients with short years of dialysis have a slow decline in physiological functions and better physiological functions. Thus, the patients have higher physiological function scores [15]. The family members of hemodialysis patients, especially the spouse, help their lives a lot, which increases the patients' motivation and confidence in overcoming the disease. Good family support can improve the patients' quality of survival and self-management ability, especially in the physiological aspect. The effect is more obvious. Therefore, it is necessary to understand the patients' family situation first and then intervene in the patients' family to improve the patients' quality of survival [16].

In the training of a conventional supervised feature representation learning network, there are various loss functions to choose from. For example, a softmax classifier can be used to obtain the category probabilities, and then, a cross-entropy loss is used to calculate the loss and train the feature extraction network [17, 18]. The cross-entropy loss is calculated as shown in equation (1), where *β* is the weight decay coefficient.

(1) $$\begin{array}{c} C_{\text{loss}}\left(x\right)=\frac{1}{n}\sum_{i=0}^{n}\left(x_{i}-1\right)+\log\frac{\beta {}^{*}\sum_{j=0}^{k}x_{j}^{2}}{2}. \end{array}$$

Transfer learning can use the knowledge learned in a domain with a sufficient calibration sample to solve a problem in another domain without a calibration sample, using the learned knowledge to solve a problem in a different but related domain. Depending on the scenario and task, the transfer learning approach varies [19]. There is a relationship between the way of using transfer learning and the amount of calibration data in the target domain and the degree of data similarity and the amount of data in the source and target domains, as shown in Table 1. Transfer learning can use the knowledge learned in the field with enough calibration samples to solve another problem in the field without calibration samples, that is, use the learned knowledge to solve problems in different but related fields. According to different scenarios and tasks, the way of transfer learning is also different.

In the metric learning model, facing the constructed metric learning-based image classification model, the contrast loss shown in equation (2) is used as the loss function based on the sample pair features calculated separately using the feature extraction network, which guides the parameter training of the feature extraction module during the optimization of the feature representation learning network, and uses the consistency constraint between similar sample pairs to improve the discriminable samples under the condition of fewer samples feature learning capability under the condition of fewer samples. The twin network uses a pair of samples *m*_*0*_, *m*_1_ as input to train the embedded feature model [20, 21]. If these two samples are from the same class *k* = 1, the distance between the obtained embedding features is small, and if these two samples are from different classes *k* = 0, the distance between the features is greater than the set threshold *m*. If it is to judge the similarity of two intervals, the commonly used measurement method is to use the commonly used European or other artificially defined distance function, which is limited to such a two-dimensional or multidimensional space, and if it is used in the case of the method proposed by Flood Sung, we broaden our thinking; we can also use neural networks to train this metric.

(2) $$\begin{array}{c} C_{\text{loss}}\left(m_{0},m_{1},k\right)=\frac{k\left|\left(f\left(m_{0}\right)-f\left(m_{1}\right)\right.\right|}{2}+\frac{\left(1-k\right)\max\left(m_{0},m_{1}\right)}{2}{\left|f\left(m_{0}\right)-f\left(m_{1}\right)\right|}^{2}. \end{array}$$

Considering that the metric learning only considers the consistency between similar sample pairs and does not have more influence on the increase of the difference between classes, this paper further uses the metric learning method of establishing similar and different class triads and uses the Triplet loss function shown in equation (3) to guide the optimal learning process of the feature representation network based on extracted features to ensure that the extracted features have good ability to portray similar images and good ability to distinguish between different classes of images under the condition of small samples. This ensures that the extracted features have a good ability to characterize similar images and distinguish between different types of images under small sample conditions [22].

(3) $$\begin{array}{c} C_{\text{loss}}\left(m_{a},m_{b},m_{c}\right)=\max\left(0,k+\left|f\left(m_{a}\right)-f\left(m_{b}\right)\right|,\left|f\left(m_{b}\right)-f\left(m_{c}\right)\right|\right). \end{array}$$

Feature dimensionality reduction refers to the selection of *N*-dimensional (*N* < *M*) features from existing *M*-dimensional features to optimize specific metrics for pattern learning tasks [23]. The main goal is to select some of the most effective features from high-dimensional feature data to reduce the dimensionality of the original feature data, which is an important means to improve the performance of pattern learning. For a pattern learning algorithm, good learning samples and effective features are the keys to train the model [24].

### 3.2. A Cognitive Computational Model of Brain Metabolism for Emotion Recognition

The flow chart of the proposed cross-individual emotion potency recognition is shown in Figure 1. Firstly, the EEG signals accompanying the emotional, cognitive activity are collected from the scalp surface of the subjects simultaneously by stimulating the corresponding emotional states with different potencies of emotional videos. Then the EEG signals are preprocessed to extract the dynamic sample entropy features and perform the feature downscaling; finally, the cross-validation strategy is used to train and test the emotion recognition algorithm and model. It is noteworthy that this paper investigates a cross-individual emotion validation method with good generalization ability, and the training data and test data used in the cross-validation strategy are based on different subjects [25]. Specifically, in the experimental study, while each subject's EEG data was used as the test data set, all other subjects' EEG data were used as the training data set. The overall performance of the proposed method is evaluated by traversing each subject in the dataset and testing the accuracy of each subject's emotional validity recognition, and then averaging the results of all subjects to obtain the accuracy of the proposed method.

When people's cognition is biased, anxiety will appear. Under the impetus of anxiety, people will further strengthen biased cognition, leading to a further increase in anxiety. In this way, the cycle of amplification will continue to increase, and the anxiety will become higher and higher, and the symptoms will increase. It is getting heavier. The sample entropy of the EEG data is extracted sequentially from a time window of width *t*_*m*_ and the duration of each movement along the time axis is ∆*t*. The sample entropy expression is defined as *S* (*x*, *y*) for an embedding dimension of *m* and a similarity threshold of *y*. Thus, for an EEG time series of time length *T*, the dynamic sample entropy expression is shown in the following equation, where the subscript *k* represents the sliding time window [26]:

(4) $$\begin{array}{c} S{\left(x,y\right)}_{k}=\sum_{i=1}^{M}s\left(x_{i},y_{i}\right)+\beta s\left(k\right),k\subseteq \left[1,M\right]. \end{array}$$

*M* in equation (1) is expressed as the number of time windows, as shown in the following equation:

(5) $$\begin{array}{c} M=\sum_{i}^{k}s\left(i\right)\left\|\frac{T-t_{m}}{\Delta t}\right\|+1-m. \end{array}$$

For the nonlinear case, as in the SVM, a kernel function is introduced to map the indistinguishable data in the low-dimensional space to the high-dimensional feature space by nonlinearity, and then the model is learned from the training samples in the new space using linear classification methods. The two classification hyperplanes of TWSVM based on the kernel function can be expressed as follows:

(6) $$\begin{array}{c} \left\{\begin{array}{c} \eta_{i}*K\left(m^{T},G^{T}\right)+\lambda_{i}=0,\;i=1,2\\ G={\left|M^{T},N^{T}\right|}^{T}+{\left|N^{T},M^{T}\right|}_{T} \end{array}\right). \end{array}$$

In dataset SEED, all subjects participated in three rounds (Sessions) of experiments, with each round spaced over 7 days apart. Each subject performed a total of 30 trials in each round, viewing one emotional video clipper trial [27]. 30 emotional video clips were played in a specific order to ensure that two video clips of the same emotional type were not presented consecutively in the experiment. Thus, dataset SEED contains EEG data samples from 30 subjects for all three emotion types, for a total of 750 EEG data samples for three rounds of experiments, with 225 EEG data samples for each emotion type. First, the EEG data were manually removed from the heavily contaminated EMG and hologram portions, and the oculomotor artefacts were directly removed from the EEG signal based on the recordings; then, the EEG data were downsampled to 200 Hz at a sampling rate of 1000 Hz. Finally, the high-frequency noise was removed using a low-pass filter from 0 to 75 Hz. The EEG data used in this study were preprocessed in the data set SEED and then subjected to some data segmentation. Specifically, the duration of each EEG data sample in the data set SEED was about 4 minutes, and only the middle part of the EEG data, the EEG data from minute 2 to minute 3 (60 seconds in total), was used in this study. EEG data from minute 2 to minute 3 (60 seconds in total) were used for the identification of emotional valence.

### 3.3. Multimodal MRI for the Therapeutic Evaluation of Maintenance Hemodialysis Patients

In this paper, a Multiparametric MRI (MP-MRI) dataset was constructed to evaluate the differentiation of HCC. Here, we refer to the images obtained by imaging modalities with different parameters as multimodal MRI imaging data, and the appearance of multimodal below refers to different kinds of MRI images. One of the most valuable MRI sequences for the diagnosis of HCC is dynamic contrast-enhanced imaging, and DCE-MRI data contain six phases, including the five periods used in the previous chapter and delayed periods. A complete six-time series of 3D stereoscopic images of DCE-MRI was used. The tumor details are more clearly presented in the color images from the fusion of multiple modal data, and the images from the fusion of data using different modalities vary, so we must combine images from multiple parameters of MRI images to more accurately assess the degree of HCC differentiation. Through experiments, we can select data with complementary characteristics for fusion to achieve better classification. When we use 2D tumor data for diagnosis, the image blocks of single modality and the image blocks of multimodal fusion can correspond to grayscale and color images in natural images, respectively, which allows us to pretrain the network on the natural image dataset and then fine-tune the pretrained model on the acquired medical image dataset for classification of medical images.

The training for the base classifier follows the structural risk minimization criterion. The structural risk minimization criterion is developed from the empirical risk minimization criterion. In pattern recognition, the error of a known sample is usually used as an estimate of the expected risk, and the risk of a known sample is called the empirical risk, which is minimized by the algorithm to pursue the minimization of the expected risk. In the three major problems of pattern recognition, the empirical risk is used as a loss function, and the empirical risk in classification is the sample misclassification rate; in the function approximation problem, the squared training error is defined as the loss function; in particular, the empirical risk minimization criterion in the probability density estimation problem is equivalent to the maximum likelihood method. The approximation of the expected risk minimum by solving for the empirical risk minimum is based on the premise that the sample data is very rich, and even under this premise, it is uncertain whether both can be simultaneously minimized. Therefore, a new criterion needs to be defined to deal with the case of a small sample size, and thus, the structural risk minimization criterion is born. Use *f*(*x*) to denote the expected risk and *P*(*f*) to denote the empirical risk obtained by the learning algorithm:

(7) $$\begin{array}{c} P\left(f\right)=\frac{\sum_{i=0}^{n}C\left(f\left(x_{i}\right)\right)}{n}. \end{array}$$

The most straightforward evaluation criterion in classification problems is Accuracy (ACC), but not only correctness is a data indicator, Sensitivity (SEN) and Specificity (SPE) are also common evaluation indicators; common curves for evaluation are subject work curves (ROC curves). The other two commonly used indicators in medicine are Positive Predictive Value (PPV) and Negative Predictive Value (NPV). The classification results are shown in Table 2.

The expressions of each indicator are shown in equation (8).

(8) $$\begin{array}{c} \left.\begin{array}{c} \text{ACC}=\frac{\left(P1+P4\right)}{\text{SUM}\left(P1,P2,P3,P4\right)},\\ \text{SEN}=\frac{P1}{\text{SUM}\left(P1,P2\right)},\\ \text{SPE}=\frac{P4}{\text{SUM}\left(P3,P4\right)},\\ \text{PPV}=\frac{P1}{\text{SUM}\left(P1,P3\right)},\\ \text{NPV}=\frac{P4}{\text{SUM}\left(P2,P4\right)}. \end{array}\right\}. \end{array}$$

Among them, the correct rate reflects the classification performance for the sample as a whole, with a higher correct rate indicating better classification performance. Sensitivity is the numerical characteristic of most interest to physicians and describes the correct classification rate for maintenance hemodialysis. The higher the sensitivity, the lower the number of maintenance hemodialysis misclassifications, and the lower the cost of this. Therefore, it is one of the most important data indicators for the classification of maintenance hemodialysis patients. The significance of specificity is the rate of correct benign classification; the higher the specificity, the lower the number of cases in which benign is misdiagnosed as malignant and unnecessary surgery is performed. These two metrics can be used to more visually represent the performance of the classification system by plotting subject work curves.

## 4. Analysis of Results

### 4.1. Model Performance Analysis

The correct rate of classification by SVM for all features is 95.15%, and the correct rate of fusion of the three classifiers using the MIN algorithm is 96.76%, and all other indicators are shown in Figure 2. The overall performance of the multiclassifier system constructed with the MIN algorithm is higher than that of the single classifier of SVM. Firstly, the sensitivity was improved. That is, the correct diagnosis rate for benign cases was higher than that of the single classifier, which could avoid unnecessary biopsies for benign patients. The specificity index of the multiclassifier system was higher than that of the single classifier, which reduced the proportion of malignant cases misclassified as benign cases and enabled more patients with malignant tumors to seek timely medical treatment and gain valuable treatment time. The positive predictive values of both classifier systems were the same. The negative predictive value of the multiclassifier system is higher than that of the single classifier, which indicates that the reliability of the malignancy classification made by the system has been further improved. In summary, the classification performance of the multiclassifier system constructed using the MIN algorithm is better than that of the single classifier trained using the SVM algorithm.

The Gauss radial basis function is chosen as the kernel function for the experiments in this paper because of its good adaptability. Therefore, the nonlinear TWSVM has three parameters, the penalty parameters C1, C2, and the Gauss kernel function related parameter *R*2 (*R* = 1/*α*2), all taking values in the range (0, 10].  Figure 3 shows the effect of the nonlinear results. It can be seen from Figure 3 that in the nonlinear case, BOA-TWSVM runs much faster than AFSA-TWSVM in both cases. According to different data sets, the test range is [20, 70]. These results show that BOA-TWSVM is effective, runs fast and robust, and outperforms other algorithms in general.

### 4.2. Computational Analysis of Brain Metabolism Cognition

Two-category cross-individual emotion validity recognition was performed based on positive and negative emotion EEG data samples from the dataset SEED. In the experimental data analysis, positive emotions were designated as positive example samples for pattern learning and negative emotions as negative example samples, and accuracy, sensitivity, specificity, and error rate were used as metrics for performance evaluation. Notably, for cross-individual emotion effectiveness identification, the training data set and the test data set were divided using the LOSO (Leave-one-subject-out) cross-validation strategy for the data set SEED. Specifically, for the 30 subjects in the dataset SEED, the experimental data of each subject is used as the test set once, while the experimental data of the other 14 subjects are all used as the training set before the test.

Figure 4 shows the results of the dynamic entropy-based EEG emotion pattern learning method for cross-individual positive and negative emotion recognition, and the experimental data results consist of the mean and standard deviation of the test results of 30 subjects. The accuracy of the dynamic entropy-based EEG pattern learning method for cross-individual positive and negative emotion recognition was 86.98%, 77.26%, and 92.98% for the EEG emotion data collected in rounds 1, 2, and 3, respectively. For the EEG data samples collected in these three rounds of experiments, the average accuracy rates of cross-individual positive and negative emotion recognition are very close, and their experimental results indicate that the dynamic entropy-based EEG emotion pattern learning approach to achieve cross-individual emotion validity recognition has good robustness.

Figure 5 gives further details of the results of the correct cross-individual positive and negative emotion recognition rates for the 30 subjects, corresponding to the accuracy of cross-individual positive and negative emotion recognition of 86.62%, 66.57%, 83.73%, 80.16%, 63.23%, 90.04%, 86.57%, 99.78%, 70.12%, 80.06%, 99.97%, 76.68%, 96.69%, 90.04% and 99.98%. The average accuracy of 89.15% is higher than the cross-individual sentiment validity recognition performance of the above single-round experiments, which is mainly due to the total sample size of 3000 for the three rounds of the dataset SEED experiments, while the sample size of the single-round experiments is only 150. In general, increasing the number of samples improves the performance of the learning algorithm, and when more sample data is used to train the learning algorithm and model, better performance of the learning algorithm can be obtained.

Figure 6 shows the relationship between the number of training and test sets of the sample sequences generated using sliding time windows of different lengths. When sample sequences are generated from EEG and speech envelope time series data using sliding time windows with data point lengths of 10, 20, 30, 40, 50, 60, 70, and 80, the numbers of training samples obtained are 480, 420, 330, 210, 140, 80, 30, and 20, respectively, and the numbers of test samples obtained are 360, 280, 250, 180, 80, 60, 24, and 15, respectively. As shown in Figure 6, for the experimental EEG data and speech envelope time series data, the shorter the window length used, the larger the number of sample sequences generated. It should be noted that the sampling rate of the preprocessed EEG data and speech envelope time series is 128 Hz, so the sample sequences with data point lengths of 10, 20, 30, 40, 50, 60, 70, and 80 correspond to 0.2 s, 0.4 s, 0.8 s, 1.2 s, 1.4 s, 1.6 s, 1.8 s, 2 s, and 2.2 s.

### 4.3. Analysis of Multimodal MRI Evaluation

The US, SWE, CEUS enhancement features, and time-intensity curves, and multimodal ultrasound all have high diagnostic value for diagnosing the benign and malignant nature of maintenance hemodialysis. The diagnostic efficacy of US, SWE, CEUS, and multimodal ultrasound for evaluating the nature of maintenance hemodialysis was compared, and the results are shown in Figure 7. The ROC curve was plotted with pathology as the gold standard, and the area under the curve of multimodal ultrasound was known to be larger by *Z* test (*P* < 0.015). The sensitivity, specificity, accuracy, positive predictive value, and negative predictive value of multimodality ultrasound were higher than those of the other three independent examinations.

Color Doppler ultrasound images provide information about the blood supply, and although they can provide blood flow information for tumor diagnosis, they have a low classification performance of 60.5% as a single basis of judgment. Electrography provides information on the hardness of the mass, which has been increasingly trusted by clinical and research staff in recent years to provide more comprehensive information for classification, with an accuracy of up to 95.6% in experiments with available data. This accuracy is obtained based on currently available data and is therefore strongly influenced by the distribution of data samples, which is difficult to achieve in practical applications. The three classifiers are used to construct a multiclassifier ensemble using the multiclassifier fusion algorithm (MIN) based on the non-Bayesian fusion framework with compound weights, and the classification results are shown in Figure 8 when compared with the improved prealgorithm (IN) without the introduction of compound weights.

## 5. Conclusion

In this paper, a cross-individual emotional validity recognition method based on dynamic entropy pattern learning is proposed. By establishing a dynamic entropy EEG pattern learning method and combining the time-course nature of mental-emotional states, we achieve the optimization of EEG emotional pattern recognition by directly representing the time-domain profile features of EEG dynamic entropy measures using entropy measure feature vectors. The cross-individual emotional state recognition was conducted on 30 experimenters using the emotional EEG dataset SEED. The experimental results show that the proposed EEG emotion recognition method achieves the best recognition accuracy of 85.12% for cross-individual positive and negative emotional states and 64.18% for cross-individual positive, neutral, and negative emotional states. The experiments fully demonstrate that the proposed emotion recognition method exhibits better generalization and generalization performance and can more effectively recognize people's mental and emotional states. According to the classification of maintenance hemodialysis by multimodal MRI, ultrasound electrography can reflect the nodule hardness and the difference in hardness with the surrounding normal tissues, and ultrasonography can show the microbleeds that cannot be detected by conventional ultrasound, which can more accurately reflect the cerebral metabolism of maintenance hemodialysis and the surrounding normal tissue perfusion status, and the combined application can provide rich and effective information for identifying the diagnosis of maintenance hemodialysis. Ultrasound-guided diagnosis has a higher accuracy rate but is an invasive test. The use of ultrasonography and shear wave electrography as auxiliary means to evaluate the nature of maintenance hemodialysis is beneficial to the qualitative diagnosis of maintenance hemodialysis, and the diagnostic value of ultrasonography for maintenance hemodialysis is improved by comprehensive analysis of all ultrasound examination indexes. The imaging omics model based on multimodal MRI plays an important role in the differential diagnosis of maintenance hemodialysis. With further in-depth research, it is expected to become a new clinically applicable objective and comprehensive diagnostic method.

## Figures and Tables

**Figure 1:** Framework for cross-individual emotional potency identification.

**Figure 2:** Comparison of classification performance.

**Figure 3:** Effect of nonlinear results.

**Figure 4:** Results of cross-individual positive and negative emotion identification.

**Figure 5:** Correct identification rate of positive and negative emotions across individuals.

**Figure 6:** Sliding time windows of different lengths versus the number of sample sequences.

**Figure 7:** Comparison between the diagnostic efficacies of each test method.

**Figure 8:** Comparison of the classification effects of MIN and IN.

**Table 1:** Applicability of transfer learning.

Data similarity	Target field data volume	Data processing method
Small	Small	Retrain several layers close to the output
Small	Big	Fine-tuned layer by layer
Big	Small	Retrain several layers close to the input
Big	Big	Retrain the model

**Table 2:** Classification results.

Serial number	Classification prediction	True prediction	Predictor
1	Benign	Benign	P1
2	Benign	Malignant	P2
3	Malignant	Benign	P3
4	Malignant	Malignant	P4

## Data Availability

Relevant data requires the consent of the corresponding author to obtain it.
